The article "Multimodality and Computational Intelligence-Enabled Intercultural Communicative Competence of College-English-Teaching Students" was retracted in 2023. Reasons: suspected computer-generated content; unreliable results or conclusions; concerns about the data; concerns about the results or conclusions.

# Multimodality and Computational Intelligence-Enabled Intercultural Communicative Competence of College-English-Teaching Students

**DOI:** 10.1155/2022/4310982

**Published:** 2022-04-28

**Authors:** Hua Zhang, Xuelin Liu

**Affiliations:** Foreign Language School, Weifang University, Weifang, Shandong 261061, China

## Abstract

With the intensification of global economic integration, international exchanges have become increasingly frequent, and employers have put forward higher requirements for ICC (Intercultural Communication Competence) of college students. In this paper, in ICC mode, the multimodal evaluation model framework of ICC is constructed by using multimodal theory. The evaluation object is Chinese college students, the evaluation media are computers and networks, and the evaluation contents include knowledge, consciousness, speculation, attitude, skills, and strategies of cross-cultural communication. The research results will help Chinese college students overcome their fears during the cross-cultural communications, meanwhile,can strengthen the cultivation of ICC for students as well. After comprehensive consideration of various influencing factors, comparing the overall teaching quality of universities of different grades or the same grade can objectively reflect the overall teaching level of the university, hoping to provide some reference for the application of multimodal discourse analysis theory and CET (college English teaching).

## 1. Introduction

According to the requirements of CET (college English teaching) reform, modern universities need to comprehensively cultivate students' comprehensive English application ability, especially strengthen the cultivation of their English listening and speaking ability, and constantly improve students' English communicative ability through various reasonable means. With the intensification of global economic integration, international exchanges have become increasingly frequent, and employers have put forward higher requirements for ICC (Intercultural Communication Competence) of college students [1]. Scientific and technological means and products are gradually involved in multimodal teaching, such as computers, multimedia, projectors, and audio- and video-recording equipment. Besides, learning related teaching techniques in combination with various other teaching methods, with the help of experience accumulation and technology, constitutes the current multimodal teaching means [2].

With the process of economic globalization, how to communicate effectively under different cultural backgrounds is becoming more and more important [3]. Economic development has put forward new requirements for people's language communication ability [4–6]. New curriculum ideas began to appear, and new language education ideas and teaching methods began to be applied in senior high school English classes. In the current all-media environment, the increasing trend of English-teaching texts is enormous, and English text abstract extraction technology is gradually applied to modern education and other fields. In practice teaching, students can have a good understanding of knowledge point [7]. This method not only plays an active role in education and teaching, such as improving teaching quality and efficiency and enriching language teaching materials, but also in cultivating intercultural communicative competence.

The article "Multimodality and Computational Intelligence-Enabled Intercultural Communicative Competence of College-English-Teaching Students" was retracted in 2023. Reasons: suspected computer-generated content; unreliable results or conclusions; concerns about the data; concerns about the results or conclusions.

There are still some shortcomings in the actual English audiovisual lectures, which limit the improvement of students' audiovisual speaking ability [8]. In the daily teaching process, teachers should balance the relationship between cultural knowledge and language knowledge learning and appropriately extend the relevant cultural knowledge in the text, such as social customs, geographical knowledge, and other humanistic knowledge so as to stimulate students' interest in English learning and cultivate students' preliminary ICC [9, 10]. This paper analyzes the problems existing in ICC training in college English at present and explores how to effectively develop ICC training in college English under the multimodal interactive teaching mode.

## 2. Related Work

Cross-cultural communication is rich in meaning, and ICC is mainly embodied in interpersonal interaction ability. Literature [11] points out that the process of cross-cultural communication is actually the process of communication and exchange by using knowledge and skills related to cross-cultural communication. Literature [12] puts forward three main aspects of cross-cultural communication, namely knowledge, purpose, and skills of cross-cultural communication. Besides, they also point out that the effect of cross-cultural communication is mainly influenced by context. Literature [13] puts forward the model of Behavior Skillpproach, which regards ICC as communicative behavior. Literature [14] further develops measurable learning results and observes the internal and external results of cross-cultural communication according to the knowledge, attitude, and skills included in ICC. Literature [15] puts forward that competence should be the evaluation of various concrete social behaviors and puts forward two criteria of ICC's social evaluation, namely, survival and appropriateness. Literature [16] points out that cultural differences often lead to two types of errors: the first is the errors of language itself, and the second is the errors of social pragmatics. Literature [17] gives a brief introduction to cross-cultural communication and other related concepts, focusing on the influence of cultural factors on people's communication, especially the communication between Chinese and Westerners, from the perspectives of linguistic and nonlinguistic means and people's communication. Literature [18] holds that ICC can be explained from three dimensions: behavior, knowledge structure, and morality. A successful communicator should have appropriate and effective behavior, relevant language and culture, knowledge of collecting information, and excellent psychological quality and, at the same time, should have a moral view of respecting and being willing to accept cultural differences. Literature [19] points out that we should pay attention to the cultivation of college students' English ICC, infiltrate cross-cultural communication knowledge in the process of high school English teaching, and use various ways to improve college students' English ICC.

The article "Multimodality and Computational Intelligence-Enabled Intercultural Communicative Competence of College-English-Teaching Students" was retracted in 2023. Reasons: suspected computer-generated content; unreliable results or conclusions; concerns about the data; concerns about the results or conclusions.

English comprehensive ability evaluation system is a complex system. With the development of systems science, management science, and scientific decision theory, a series of theories and methods of systematic analysis and decision-making have emerged correspondingly. The evaluation forms mainly include peer evaluation and student evaluation. This kind of teaching quality evaluation method has been widely used in universities and achieved certain results. Literature [20] empirical research shows that there are six characteristics that can explain the variation of 25.8% of students' evaluation results, and students' evaluation of teachers' teaching has certain limitations, which can only be used as a reference for teachers to improve teaching. Literature [21] proposes to discuss senior high school English vocabulary teaching from the perspective of ICC cultivation and proposes that senior high school English vocabulary teaching should be combined with cultural context to better improve the teaching effect of vocabulary teaching, and the combination of ICC cultivation and textbook research should be infiltrated into vocabulary teaching. Literature [22] puts forward an effective way to cultivate students' ICC by analyzing the cross-cultural ideas embodied in Oxford English textbooks. Literature [23] proposes to cultivate students' English ICC in the process of language skills training. Literature [24] puts forward an effective way to cultivate students' ICC based on core literacy. Literature [25] puts forward that ICC training should be combined with local culture to better cultivate students' initial ICC.

The article "Multimodality and Computational Intelligence-Enabled Intercultural Communicative Competence of College-English-Teaching Students" was retracted in 2023. Reasons: suspected computer-generated content; unreliable results or conclusions; concerns about the data; concerns about the results or conclusions.

In the process of cultivating students' cross-cultural communication ability, we should pay attention to the changes in students' thinking and psychology. By paying attention to students' nonintelligence factors, it is necessary to timely and effectively adjust the teaching methods and training programs of cross-cultural communication so that students can truly participate in English class, experience the differences between Chinese and western cultures, make students become masters of learning, be able to master the cultural knowledge they have learned, and learn to communicate with people from different cultural backgrounds in different scenes.

## 3. Research Method

### 3.1. Investigation on ICC of College Students in English

When implementing multimodal audiovisual lectures, teachers should coordinate the application of the two modes reasonably and maximize the advantages of the two modes. On the one hand, with the help of visual modality, it is necessary to effectively supplement the auditory modality. While ensuring the clarity of visual modality information, with the help of visual advantages, it is necessary to complement the incomplete auditory content and ensure the effective degree of information. On the other hand, use hearing to visualize visual content, ensure the intuitiveness and vividness of the information, and arouse students' emotional resonance so that they can get a better audiovisual training experience.

The subjects of this study are 390 freshmen in a university. The researcher randomly selected five classes of freshmen in an internship school to conduct a questionnaire survey. The reason why freshmen are selected as the survey object in this survey is that freshmen's schoolwork burden is relatively small, they can have a certain amount of time to cooperate with the survey, the survey is highly operational, and the authenticity of the data can be guaranteed.

In order to provide more substantial materials for this research, it can also make the research more convincing. In this study, an interview was conducted with English teachers of freshmen. Five teachers have been teaching for 3 to 7 years, and their ages range from 35 to 45 years. One was a male teacher, and four were female teachers. The interview content is as follows:

1. How much do you care about cross-cultural communication knowledge in English teaching, and why?
2. Do you think that learning cross-cultural communication knowledge will help students improve their self-confidence in learning English and improve their grades?
3. In the teaching process, do you introduce western cultural background knowledge suitable for the text to students? If so, what are your practices?
4. What methods do you usually use to cultivate students' ICC?

The article "Multimodality and Computational Intelligence-Enabled Intercultural Communicative Competence of College-English-Teaching Students" was retracted in 2023. Reasons: suspected computer-generated content; unreliable results or conclusions; concerns about the data; concerns about the results or conclusions.

English curriculum standards require students' ICC and awareness. How do you understand this requirement?

This study adopts the methods of literature research, questionnaire survey, and interview, and with the help of test paper, questionnaire, and interview outline, it studies the current situation of ICC in college English. The test questionnaire used in this study is ICC self-test scale. Cross-cultural communication self-test scale includes five test elements, namely, language competence, strategy competence, cross-cultural knowledge, cross-cultural attitude, and cross-cultural awareness.

This scale uses five figures to investigate, and “1” indicates noncompliance or basic noncompliance, which rarely accords with your actual situation. “2” means that it is usually not in conformity with the actual situation, and the probability of this expression being in conformity with the actual situation is less than half. “3” means to a certain extent, and the expression conforms to the actual situation in half of the cases. “4” is usually quite consistent, and the probability that this expression conforms to the actual situation is more than half. “5” means always or basically in line with, and this expression basically conforms to the basic situation, that is, 100% (Figure 1).

Situational teaching is an effective means of audiovisual and speaking teaching. At present, the interaction time between teachers and students in English teaching is relatively small, and the time left for students to think and speak is relatively small, which will limit the implementation of situational teaching mode. In interpersonal communication, it is necessary to communicate with the above five modes, so communication is a multimodal activity.

Cross-cultural communication needs language, images, sounds, behaviors, and other means and symbols, and at the same time, it also needs the cooperation of the five senses. This communicative ability can be exercised in the process of learning a foreign language, but it does not just come from this, so the foreign language level cannot be directly equated with communicative ability. Foreign language teaching consciously influences students, cultivates cross-cultural communication awareness, and cultivates and exercises cross-culture.

Modern educational technology and rich teaching resources provide rich teaching means for CET, create more convenient conditions for CET, and provide a broader teaching space. Just as CET should not only pay attention to the cultivation of listening, reading comprehension, writing, and other abilities, CET should also be carried out in many ways, and single-mode CET cannot achieve the best teaching effect. CET is not only to comprehensively train students and cultivate their comprehensive quality but also to comprehensively stimulate their senses, stimulate their learning potential, and realize effective CET [1].

The article "Multimodality and Computational Intelligence-Enabled Intercultural Communicative Competence of College-English-Teaching Students" was retracted in 2023. Reasons: suspected computer-generated content; unreliable results or conclusions; concerns about the data; concerns about the results or conclusions.

### 3.2. Cultivation of ICC in College English under Multimodal Teaching Mode

Cross-cultural communication is not a general term, which includes three basic elements: cross-cultural communication, cross-cultural awareness, and strategies and methods used in cross-cultural communication. This concept also has a high degree of recognition in academic circles. Multimedia-specific dynamic videos and audio guide students so that they can better understand the cultural meaning and connotation of language symbols, and the current situation that college students lack the ability of cross-cultural communication will not be caused.

From the perspective of cultural popularization, language teaching and practice can not only consolidate and strengthen students' ability to master and apply language but also cannot lead students to share movies and television as a kind of fun. Not only is language teaching not done well but also students' ability of cross-cultural communication is not cultivated. For example, imitating the plot in groups, performing sitcoms, and describing and continuing the content of the film can help students to better perceive the ethics and cultural details in the film and master the application ability while learning the language.

Whether it is the story in a literary work or the picture depicted, when combined with the language of the characters in the picture, it gives life to the work, which makes the readers have an immersive sense of life. For another example, if the teaching content has various modes of sound, words, images, and even different colors and fonts, it can activate students' various senses and fully integrate various symbol resources such as images, sounds, and words, thus deepening learners' impression and improving their memory ability and making the teaching effect much better than simple language explanation.

As an important evaluation method, the content and means of testing cannot be specified out of thin air but should be consistent with teaching objectives and teaching methods. First, select the appropriate teaching method according to the teaching environment (including teaching purpose, content, and object) and then select the appropriate teaching mode. According to the principle of consistency of teaching evaluation, the evaluation mode is consistent with the teaching mode as shown in Figure 2.

In the author's evaluation model, the teaching object is college students, the teaching purpose is to cultivate and improve college students' ICC, and the complete teaching content includes six aspects of cross-cultural communication knowledge, consciousness, speculation, attitude, skills, and strategies. Under the guidance of this overall goal and content, specific teaching methods and teaching modes involve more specific teaching designs and arrangements. According to the principle of teaching students in accordance with their aptitude, first of all, students and teaching contents should be graded and layered. For different teaching contents and teaching objects, teaching methods and teaching modes are different.

The article "Multimodality and Computational Intelligence-Enabled Intercultural Communicative Competence of College-English-Teaching Students" was retracted in 2023. Reasons: suspected computer-generated content; unreliable results or conclusions; concerns about the data; concerns about the results or conclusions.

Using the closeness formula of spatial distance and human brain cognition in attribute theory, let the score of a school in the *i*th grade be *X*(*x*_1_, *x*_2_,…, *x*_*n*_), and its satisfaction degree be [3]

(1) $$\begin{array}{c} C_{s}\left(X\right)=\exp\left(-\left(\frac{\sum_{i=1}^{n}w_{i}\left|x_{i}-y_{i}\right|}{\sum_{i=1}^{n}w_{i}\delta_{i}}\right)\right). \end{array}$$

The satisfaction degree of the same grade is obtained by the formula of closeness degree (1), but the standard points of satisfaction are different among different grades, so when calculating the satisfaction degree, the reference standard points are also different. Therefore, according to the satisfaction degree calculated now, it is still difficult to compare the quality of schools in different grades according to the degree to which they meet the standards. Namely,

(2) $$\begin{array}{c} C_{t}=\left(X\right)\\ =\lambda C_{s}\left(X\right). \end{array}$$

Among them, *C*_*s*_(*X*) is the grade satisfaction of school *X*; *λ* is related to the total score of school *X*. *λ*=*f*(∑*x*_*i*_) and *x*_*i*_ are the *i*th attribute scores of school *X*. Here, select a *λ*.

(3) $$\begin{array}{c} \lambda ={\left(\frac{\sum x_{i}}{\text{full marks}}\right)}^{\alpha },\;\alpha >0. \end{array}$$

The coefficient *α* can be adjusted according to the actual effect.

The query vector set is integrated with the query interface, the hidden information transmission channel and feature extraction module, and the English article query information output module to construct the distributed storage of English articles, and the ontology model of English text abstract is constructed by using triples, which is shown in the following formula:

(4) $$\begin{array}{c} C=\min\left\{\max\left(C_{i}\right)\right\},\\ \sum_{j^{\prime }=1}^{p^{\prime }}Z_{i,j,j^{\prime }}=1,\;\forall_{i}\in \left(1,n\right),\;\forall_{j}\in \left(1,n_{i}\right). \end{array}$$

According to the English article ontology model, the Wigner–Ville spatial distribution of English text abstract database is constructed, and the information flow characteristics of different sampling time intervals are obtained in Wigner–Ville space.

The article "Multimodality and Computational Intelligence-Enabled Intercultural Communicative Competence of College-English-Teaching Students" was retracted in 2023. Reasons: suspected computer-generated content; unreliable results or conclusions; concerns about the data; concerns about the results or conclusions.

The limited English text abstract set *X* is divided into class *C*, and the formation direction of semantic ontology vectors in English abstracts has *M* direction sets. By preprocessing and screening English abstracts, the overall structure of English abstract extraction in English teaching is obtained.

According to the result of probability density distribution, the extraction rate of each phase point in the region can be obtained as shown in the following formula:

(5) $$\begin{array}{c} Q_{w}\left(\omega \right)=\frac{\sum K_{wpg}\left(W_{pg}\right)}{p\times q}. \end{array}$$

The confidence space of the distribution effectiveness of English time-frequency distribution feature points is shown in the following formula:

(6) $$\begin{array}{c} \sum_{i=1}^{c}\mu_{ik}=1,\;k=1,2,\cdots ,n. \end{array}$$

Therefore, finally, the clustering function of English text summary information is optimized, and English text summary extraction based on semantic feature points of English text summary is realized.

## 4. Results Analysis and Discussion

In today's college English class, more and more teachers choose to use multimedia projection to teach students, while blackboard writing is less and less used. According to observation and research, it can be found that the teaching mode of “text + multimedia network technology + teacher guidance” can better arouse students' interest in learning and then improve their language ability. However, while making full use of tool teaching, it lacks the embodiment of language humanity.

On the aspect of cross-cultural knowledge, questions 24 and 25 show that freshmen can respond correctly, pay attention to their self-image, and keep a suitable social distance when dealing with people of different cultures (Figure 3).

Through the analysis of cross-cultural knowledge, it can be seen that most students pay attention to their dress and image when communicating and can understand the appropriate communication distance in each other's culture. In the cross-cultural communication questions, from questions 27 to 32, it can be seen that students do not know the historical figures and events of English-speaking countries' culture, and they do not know the literary works and important writers in English culture.

Due to the teaching environment in China and the design of CET, it is difficult for CET to actually train students' ICC. Many CETs are offered for a short period of time, with fewer courses, and many English courses are specialized English teaching based on related majors, which are somewhat restrictive in content.

The article "Multimodality and Computational Intelligence-Enabled Intercultural Communicative Competence of College-English-Teaching Students" was retracted in 2023. Reasons: suspected computer-generated content; unreliable results or conclusions; concerns about the data; concerns about the results or conclusions.

Through the cross-cultural attitude test, only 113 students are interested in different thinkings in other countries and willing to communicate with people from different cultures (Figure 4).

Through the above analysis, it can be seen that most students lack the initiative of communication, and only 113 students are willing to communicate with people from different cultures. There are 176 people who cannot respond actively. It can be seen that most freshmen are very concerned about English cultural phenomena, hoping to learn more about the social and cultural knowledge of English-speaking countries. Be able to consider for others when communicating.

Students must receive the infection and edification of humanistic thoughts by reading newspapers, novels, and other different types of texts to cultivate their English intercultural communicative competence. Therefore, teachers should recommend suitable reading materials for students on the basis of understanding students' cognitive ability, reading level, interests, and needs. In the world of extracurricular reading, students gain not only language knowledge and language skills but also broader cultural background knowledge and more speculative learning thinking. The statistical results of cross-cultural awareness are shown in Figure 5.

It can be seen that freshmen think that the purpose of learning English is to cope with exams, not to learn English cultural knowledge and cultivate English ICC. In the process of communication, students cannot adjust their communicative behavior flexibly. At the same time, most students find it difficult to adjust their communicative behavior according to the cultural background of both sides.

First-year teachers will use group learning to explain the cultural background knowledge and cross-cultural communication knowledge related to the text. Before class, they will divide groups and assign tasks so that students can consult materials and form reports. In class, they will evaluate the results of group learning by showing the results of group learning and point out the shortcomings. For example, when it comes to the way of communication in the UK, teachers often ask students to play specific roles to have situational dialogues to understand the social habits in the UK. At the same time, the teacher will let the students know the differences between Chinese and Western cultures by comparing our ways of communication with those of British people.

Generally speaking, in the way of explaining cross-cultural communication knowledge and text background cultural knowledge, three teachers will explain relevant cultural background knowledge through case analysis in classroom teaching. Before class, the teacher will assign homework for group study, form a reading report by consulting relevant materials, and share the results in class to learn the cultural background knowledge of the text. In addition, the teacher will directly explain the cultural knowledge in the test questions and homework and help improve students' reading comprehension of the text.

The article "Multimodality and Computational Intelligence-Enabled Intercultural Communicative Competence of College-English-Teaching Students" was retracted in 2023. Reasons: suspected computer-generated content; unreliable results or conclusions; concerns about the data; concerns about the results or conclusions.

Only a few teachers will teach English cultural knowledge in various forms such as group learning. Generally, freshmen mainly learn English cultural knowledge through teachers' direct explanation of the cultural background knowledge involved in textbooks or exam reading questions, and English cultural knowledge is mainly learned through after-class reading exercises. At the same time, due to the relatively heavy schoolwork burden of students, students rarely have time to learn English cultural knowledge by watching movies, extracurricular books, and other forms, so the way for students to learn English cultural knowledge is relatively simple.  Figure 6 shows the evaluation results of CET comprehensive ability.

Teachers can first introduce that in our culture, Chinese is subjective and comprehensive and advocate combining the subject with the world to know the world and pay more attention to expressing inner feelings. The meaning of Chinese expression is less dependent on form, while western culture advocates understanding the world with an accurate and objective attitude, so western language is more accurate and profound, and grammatical expression is also more accurate. Through learning the above cultural background knowledge in classroom teaching, students will pay more attention to the differences between Chinese and Western language expressions.

Based on this advantage of multimodal interactive teaching, many universities have introduced modern technologies such as multimedia, projector, and computer into English teaching, in order to provide students with multidimensional and multisensory information forms, thus improving classroom teaching efficiency and English teaching quality. The statistical data indicators of each node can further and quantitatively reflect the actual influence effects of various factors (as shown in Figure 7).

It is not difficult to find that the foundation of English for admission is generally not as high as that of “Happy English” and “High Starting Point,” especially in listening and speaking. Therefore, this group of students relies heavily on computer-assisted teaching tools such as multimedia teaching. For this kind of students, in particular, it is necessary to strengthen the use of multimedia teaching tools and develop high-quality teaching courseware covering “listening, speaking, reading, and writing.”

The article "Multimodality and Computational Intelligence-Enabled Intercultural Communicative Competence of College-English-Teaching Students" was retracted in 2023. Reasons: suspected computer-generated content; unreliable results or conclusions; concerns about the data; concerns about the results or conclusions.

Through a large number of English text abstracts, the quality of English teaching and the sharing of English teaching resources can be improved. It can extract the well-distributed features of text data in English articles and realize the classification and management of features. On this basis, it can get the key content classification and text features that we have learned and mastered.

Therefore, the extraction of English text abstracts is the basis of optimizing teaching and reading English articles quickly [2–4]. According to the simulation parameter settings, compared with the algorithms in [22, 23], the extraction accuracy results are shown in Figure 8.

In Figure 2, the analysis results show that the accuracy of this method for English text abstract extraction is better than the other two algorithms. From the detail point of view, with the increase in iteration times, the accuracy is also constantly improving. The proposed method only needs 14 iterations to achieve 100% accuracy, while the algorithm in reference [22] needs about 20 iterations.

With the change of the new curriculum standards, the compilation of new textbooks also fully takes into account the importance of English cultural knowledge teaching and makes English cultural knowledge teaching an important part of college English teaching. For example, in the new version of the People's Education Edition English textbook used by freshmen in practice schools, there are many texts of English culture categories. Based on this situation, teachers should make full use of the existing English classes, comprehensively sort out and integrate the cultural information in the textbooks according to the existing new textbooks, and teach students English cultural knowledge more comprehensively and systematically.

Universities do not pay enough attention to the cultural communication function of language, but they are relatively deficient in cross-cultural knowledge. In fact, many modern tools provide abundant resources for language teaching. If students only learn about cross-cultural knowledge from texts or teachers' mouths, the content they master will be greatly limited, even with certain prejudice. Taking the extracted speed as the test index, the simulation comparison results are shown in Figure 9.

The results show that this method can achieve convergence in a short time, which indicates that this method has good convergence and real-time performance.

Through the creation of pragmatic situations and the setting of oral exercises, every student should participate in practical exercises as much as possible so as to accumulate experience and sum up skills through practical training. Teachers can divide students into several groups, role-play the video content, restore the scene, and evaluate the performance of groups and students, focusing on the performance related to language communication such as students' pronunciation, intonation, and grammar so as to help students understand the loopholes in their own learning process and thus make learning targeted.

The article "Multimodality and Computational Intelligence-Enabled Intercultural Communicative Competence of College-English-Teaching Students" was retracted in 2023. Reasons: suspected computer-generated content; unreliable results or conclusions; concerns about the data; concerns about the results or conclusions.

Through the questionnaire, it is found that the CET of the junior year where the internship school is located lacks various forms of English practice activities, and students are only exposed to English through the basic forms of classroom learning. In view of this situation, teachers can use various forms of activities to stimulate students' interest in learning English cultural knowledge, for example, before the new knowledge is taught, they can use 3–5 minutes to introduce some cultural background knowledge related to the text so that students can express their views and opinions. In addition, teachers can hold various English practice activities after class. For example, when learning Unit 5 Language and Characters, teachers can ask students to collect some information about the differences between Chinese characters and western characters, exchange and share the results in the form of theme class meetings, and better cultivate students' ICC by learning this unit.

In short, teachers should strengthen the research and application of various teaching modes; make good use and combination of visual, auditory, and tactile modes; and constantly enrich their own modal teaching methods to ensure the effectiveness and interest of visual, listening, and speaking teaching.

## 5. Conclusion

On the basis of multimodal teaching theory, this paper advocates that the ICC of college students at different levels should be tested by using text mode, image mode, hearing mode, body mode, and their reasonable combination. In CET, first of all, students should master and be familiar with using language points and skills and then step into culture teaching with the help of language teaching so that students can deeply feel the charm and connotation of foreign culture and cultivate students' ICC thinking and perception. This requires that ICC should be cultivated from the student period. In writing class, students need not only written practice but also oral practice. Teachers should first let students use the sentence patterns they have learned in class for expression training. By combining with the context, students can really enrich their corpus and learn to use more sentence patterns and rich vocabulary for oral communication and written writing practice.

The article "Multimodality and Computational Intelligence-Enabled Intercultural Communicative Competence of College-English-Teaching Students" was retracted in 2023. Reasons: suspected computer-generated content; unreliable results or conclusions; concerns about the data; concerns about the results or conclusions.

## Figures and Tables

**Figure 1:** Classification of college students' cross-communication ability self-test scale.

**Figure 2:** Basic ideas of ICC multimodal evaluation.

**Figure 3:** Intercultural knowledge.

**Figure 4:** Cross-cultural attitude.

**Figure 5:** Cross-cultural awareness.

**Figure 6:** Evaluation results of comprehensive ability of CET.

**Figure 7:** Statistical data indicators of some nodes.

**Figure 8:** Comparison of accuracy of text abstract extraction in English teaching.

**Figure 9:** Convergence test of root mean square error normalization.

## Data Availability

The data sets used and/or analyzed during the current study are available from the corresponding author on reasonable request.
